The article "Indoor Acoustic Signals Enhanced Algorithm and Visualization Analysis" was published in 2021. Journal: Comput Intell Neurosci.

# Indoor Acoustic Signals Enhanced Algorithm and Visualization Analysis

**DOI:** 10.1155/2021/7592064

**Published:** 2021-07-31

**Authors:** Suqing Yan, Xiaonan Luo, Xiyan Sun, Jianming Xiao, Jingyue Jiang

**Affiliations:** ^1^School of Information and Communication, Guilin University of Electronic Technology, Guilin 541004, China; ^2^Guangxi Key Laboratory of Precision Navigation Technology and Application, Guilin University of Electronic Technology, Guilin 541004, China; ^3^Guangxi Key Laboratory of Image and Graphic Intelligent Processing, Guilin University of Electronic Technology, Guilin 541004, China; ^4^National & Local Joint Engineering Research Center of Satellite Navigation and Location Service, Guilin University of Electronic Technology, Guilin 541004, China; ^5^Guilin University, Guilin 541004, China

## Abstract

A pure acoustic signal can be easy to realize signal analysis and feature extraction. However, the surrounding noises will affect the content of acoustic signals as well as auditory fatigue to the audience. Therefore, it is vital to overcome the problem of noises that affect the acoustic signal. An indoor acoustic signal enhanced method based on image source (IS) method, filtered-x least mean square (FxLMS) algorithm, and the combination of Delaunay triangulation and fuzzy c-means (FCM) clustering algorithm is proposed. In the first stage of the proposed system, the IS method was used to simulate indoor impulse response. Next, the FxLMS algorithm was used to reduce the acoustic signals with noise. Lastly, the quiet areas are optimized and visualized by combining the Delaunay triangulation and FCM clustering algorithm. The experimental analysis results on the proposed system show that better noise reduction can be achieved than the most widely used least mean square algorithm. Visualization was validated with an intuitive understanding of the indoor sound field distribution and the quiet areas.

## 1. Introduction

An acoustic signal is the most widely used signal in real life. However, there is a lot of noise that disturbs the original acoustics signal. Excessive environmental noise harms people's physiological and psychological health [1]. Furthermore, long-term exposure to a high noisy environment will cause serious harm to people's health and affect their daily life [2]. Statistics show that more than 70 percent of the world's urban residents are affected by noise pollution [3]. And it is difficult to communicate with people in noisy environments. Even the phenomenon that you cannot hear or not hear clearly occurs. Therefore, acoustic enhancements have caused growing concern all over the world.

Acoustic enhancement algorithms include commonly spectral subtraction, wiener filtering, and adaptive filtering. Boll proposed firstly the spectral subtraction algorithm with low computational complexity and easy implementation [4]. However, the music noise is caused for nonlinear processing of inaccurate amplitude estimation, and the speech roughness was produced for the lack of phase information of the pure signal. Then, Berouti et al. proposed nonlinear spectral subtraction [5], Gustafsson et al. proposed adaptive gain average spectral subtraction [6], and SIM et al. proposed minimum mean square error spectral subtraction [7]; these methods are not perfect. Lim and Oppenheim [8, 9] proposed the wiener filtering algorithm of speech enhancement. The premise of the wiener filtering is that the speech can be calculated by the AR model. Then, the noise can be reduced by estimating the AR parameters of pure speech. Compared with spectral subtraction and Wiener filtering methods which require prior knowledge of noise and pure acoustic signals, adaptive filtering methods can dynamically adjust filter parameters using adaptive algorithms under unknown noise conditions to ensure optimal noise suppression performance. Therefore, noise reduction algorithms based on adaptive filtering have been widely used.

The article "Indoor Acoustic Signals Enhanced Algorithm and Visualization Analysis" was published in 2021. Journal: Comput Intell Neurosci.

Active noise reduction methods eliminate the noise mixed in the useful signal using an adaptive algorithm, adjusting the parameters adaptively [10, 11]. This method is widely used due to its lower complexity and better controllability. Among the active noise reduction algorithms, the least mean square (LMS) algorithm is classical adaptive algorithms [12, 13]. However, due to the fact that its fixed-step manner slowly reaches the optimal coefficient of the whole system, the convergence speed of the LMS algorithm is relatively slow. As a result, the noise cannot be processed and analyzed in real time. Therefore, the filtered-x least mean square (FxLMS) algorithm can eliminate both high- and low-frequency noises [14, 15]. Furthermore, when the error between the received noise and the expected residual becomes more significant, the step is increased to accelerate its convergence to the wiener solution and vice versa.

There are three indoor acoustic simulation methods: wave acoustic method, statistical acoustic method, and geometric acoustic method [16]. The wave acoustic method focuses on studying the effect of standing wave resonance in the room by wave theory [17]. Craggs proposed the finite element method [18] based on the wave acoustic theory. Kopuz and Lalor proposed the boundary element method [19], and Botteldooren proposed the time-domain finite difference method [20]. The statistical acoustic approach focuses on measuring the energy, ignoring the acoustic wave characteristics [17]. Forssen et al. proposed the statistical energy analysis (SEA) to realize the sound field in the railway [21]. The geometric acoustic method ignores acoustic wave characteristics and uses sound lines to describe the sound propagation path when studying the free sound field's diffusion. Krokstad et al. proposed the ray tracing method (RTM) [22]. Allen and Berkley proposed an image source method based on geometric acoustics [23]. Finally, Vorlander combined the tracking method with the image source method [24] to improve the efficiency and accuracy of the indoor acoustic simulation.

The article "Indoor Acoustic Signals Enhanced Algorithm and Visualization Analysis" was published in 2021. Journal: Comput Intell Neurosci.

The wave-based method is limited to some specific situations, which are used in a small room with uneven frequency distribution and less resonant frequency in low frequency. In addition, the statistical acoustic method is suitable for high frequency and large-sized space. The geometric acoustic method ignores the acoustic fluctuation and is applicable when the indoor sound propagates to an interface whose size is much larger than the sound wavelength. Among the methods mentioned above, the geometrical method has both high accuracy and more applications. The image source (IS) method is the most typical geometrical acoustic method, and it has been widely used in practical applications [25, 26].

In indoor environments, unreliable prior knowledge between noise and pure acoustic signals, and difficult-to-estimate noise degrade the performance of acoustic enhancement and pose great challenges for attaining the pure acoustic signals. Aiming at a better performance on acoustic enhancement, we propose a novel indoor acoustic signals enhanced method. The basic idea of this method is to produce adaptively the reverse signal equal to the external noise, then to get pure signal by the addition of the received signal and the reverse signal. Finally, the quiet areas are optimized and visualized by combining the Delaunay triangulation and FCM clustering algorithm. The main contributions in this paper are as follows:

  Noise reduction based on the FxLMS algorithm is presented for indoor spatial structure. The comparison between the FxLMS algorithm and the LMS algorithm has been researched for noise inhibition of indoor environments. The results demonstrate that the performance of the noise reduction based on the FxLMS algorithm has dramatically improved.
  We propose to adopt the Delaunay triangulation and FCM clustering algorithm to analyze the acoustic signal and visualize noise inhibition in indoor environments. The visualization demonstration of noise inhibition is more conducive to examining the indoor effect and specific distribution of indoor noise reduction.

The article "Indoor Acoustic Signals Enhanced Algorithm and Visualization Analysis" was published in 2021. Journal: Comput Intell Neurosci.

The remainder of this article is arranged as follows. In Section 2, we discuss noise reduction and the visualization of acoustic field distribution. The proposed method is introduced in Section 3 including the FxLMS algorithm and FCM clustering algorithm. Experimental results are depicted in Section 4. Finally, the conclusions are summarized in Section 5.

## 2. Related Work

### 2.1. Noise Reduction

Active noise reduction is realized with superposition and cancellation of the controlled acoustic wave and original noise. It can effectively suppress low-frequency noise that is difficult to reduce in the passive method.

The FxLMS algorithm is an active noise control method. The secondary channel composed of a loudspeaker and error sensor is used in the FxLMS algorithm [15, 27]. The input reference signal is processed to get the control signal. The weight vector of the FxLMS algorithm is modified by comparing the control signal with the error signal so that it can be adjusted at all the target frequency bands. Erkan completed the headset design of a single channel, which is realized by the FxLMS algorithm [28]. Liu analyzed the performance of a narrow-band active noise control system based on the FxLMS algorithm [29]. Kuo researched the FxLMS algorithm on an embedded platform [30]. Jordan and Elliott constructed a multichannel FxLMS active noise reduction system to suppress the multiline spectrum superimposed noise generated by the yacht engine and proposed a method to determine the convergence coefficient of each channel [31].

### 2.2. Noise Inhibition Visualization

Visualization is an intuitive method to help researchers know acoustic fields. However, visualizing acoustic fields is a complex problem in the acoustic simulation since sound will incur the reflection and absorption during the propagation. Oikawa et al. described the united visualization for acoustic field and the source fluctuation using the 3D laser [32]. Acoustical holography is the most widely used acoustic visualization technology. Wang and Bei applied an optimization method in the design of a microphone array [33]. Koprinkova-Hristova and Alexiev proposed a dynamic visual approach for acoustic camera perception [34] and created a 3D visualization of acoustic wave propagation in time. To visualize acoustic fields, the sound is typically estimated using active noise control (ANC) in the room at a given time in this paper; the sound field distribution during propagation and the quiet areas after noise reduction is visualized.

## 3. Proposed Method

In this section, a novel indoor acoustic signal enhanced method is proposed, aiming to realize a better performance for noise reduction and the conducive visualization of the acoustic signal distribution. The framework of our proposed method includes three stages. In the first stage, a reverberation acoustic signal is simulated by the IS method. Then, the reverse signals equal to the noises are produced by the FxLMS algorithm, and the denoised signal is gained by the addition of the reverberation signals and the reverse signal. After noise reduction, the data can be divided into different subsets. Then, all the quiet points are clustered through the FCM clustering algorithm. We adopt the Delaunay triangulation to subseparate the quiet points set. Lastly, visualization is developed for indoor acoustic signal distribution and the quiet areas in the room.

The article "Indoor Acoustic Signals Enhanced Algorithm and Visualization Analysis" was published in 2021. Journal: Comput Intell Neurosci.

### 3.1. Acoustic Signal Simulation

In this paper, the source acoustic signal is recorded by the audiorecorder function of MATLAB, its sampling frequency fs = 8000 Hz, and the format is audio1 = audiorecorder (8000, 16, 1). The IS method [23] is adopted to simulate the impulse response in indoor environments. Therefore, the acoustic simulation results of the received position in the space can be obtained.

In indoor environments, the sound may be reflected in each wall. Therefore, an image sound can be considered at each reflection. The distributions of the sound source and image source and the received position in 3D space are shown in Figure 1. *S* and *R* denote the sound source position and the received position, respectively. *S*1, *S*2, *S*3, and *S*4 are the image source positions. In Figure 1(b), a solid arrow represents the direct path between the source position *S* and the received position *R*, and reflected paths between the image source positions and the received position *R* are represented by the dotted arrow.

Suppose the virtual room is *a∗b∗c*, the received position $R=\left[\begin{array}{ccc} R_{x} & R_{y} & R_{z} \end{array}\right]$, and the source position $S=\left[\begin{array}{ccc} S_{x} & S_{y} & S_{z} \end{array}\right]$. Only analyze two boundaries *y* = 0 and *y* = *b* for simplicity without loss of generality. The two image positions will be $S_{1}=\left[\begin{array}{ccc} S_{x} & -S_{y} & S_{z} \end{array}\right]$ and $S_{2}=\left[\begin{array}{ccc} S_{x} & 2b-S_{y} & S_{z} \end{array}\right]$, and the distances from *S*1, *S*2 to *R* can be computed. We can also obtain the other image source positions and calculate the distances in the same way; the impulse response of the room is obtained by the image source (IS) method. Therefore, the total acoustic signals of the received position should be gained by the acoustic and all reflected acoustics in the received position.

The article "Indoor Acoustic Signals Enhanced Algorithm and Visualization Analysis" was published in 2021. Journal: Comput Intell Neurosci.

As a result, the sound will be reflected in each boundary, and image sound can also be propagated and reflected at each border. The number of image sounds will increase exponentially, and the calculation will be much more complex with multiple reflections considered. However, the farther the image sounds are from the received position, the more the attenuation will be. It is crucial to analyze the reflected distribution for simulating indoor sound with more accuracy. Given *K* be the number of reflections, let *k* be [−*K: K*].

Therefore, the array composed by image acoustic signal path can be expressed as follows:

(1) $$\begin{array}{c} M_{k}=k+0.5*\left[1+{\left(-1\right)}^{k}\right]. \end{array}$$

After determining all image positions, the distance from the source position *S* to the received position *R* is presented as

(2) $$\begin{array}{c} D_{k}=\left|{\left(-1\right)}^{k}*S+M_{k}*M-R\right|, \end{array}$$

where *M* denotes room position. Sound signals of the received position are got if multiple acoustic signals arrive at the received position.

The acoustic signal must be convolved to get acoustic fluctuation at the received position. The convolution is represented as

(3) $$\begin{array}{c} G\left(k\right)=\sum_{j}Q\left(j\right)\varphi \left(k-j+1\right), \end{array}$$

where *Q* is the source data after normalization and *φ* is the spatial impact factor vector. Then, the indoor image acoustic signal simulation model can be expressed. The signal *G* can be obtained by the convolution of the function *φ* and the source signal *Q*. Hence, the final output *G* is the fixed-point acoustic simulation result of the received position under the condition of indoor space based on the image source method.

To simulate the acoustic signal in the indoor environment, we suppose that the parameters as follows: room size is 5 × 7 × 3 m^3^, the boundary of the walls is not rigid, the absorption coefficient is 0.4, acoustic source position is *S* = [0.5 0.5 2.5] *m*, and reflection coefficient $K=\left[\begin{array}{ccc} 0 & 5 & 15 \end{array}\right]$.

Figure 2 shows the simulation results with different received positions. The distance *D*1 from the source position S to received position *R*1 = [3.5 5.0 1.3] m is *D*1 = 5.5399 m, the distance *D*2 from the source position *S* to received position *R*2 = [2.0 3.0 1.3] m is *D*2 = 3.1528 m, and the distance *D*3 from the source position *S* to received position *R3* = [0.5 5.0 1.3] m is *D*3 = 4.6573 m. Then, the signal reaches the received positions *R*1, *R*2, *R*3 at [129, 74, 109] as shown in Figure 2(a) at *K* = 0.

### 3.2. FxLMS Algorithm

FxLMS algorithm [14] structure is shown in Figure 3. In Figure 3, *P*(*z*), *S*(*z*), and $\hat{S}\left(z\right)$ are the transfer function of the primary path, the secondary path, and the secondary path model, respectively. The desired signal *d*(*n*) is the output signal of the primary path. The coefficient of the secondary path is controlled by the residual noise or error signal *e*(*n*) that minimizes the noise.

The article "Indoor Acoustic Signals Enhanced Algorithm and Visualization Analysis" was published in 2021. Journal: Comput Intell Neurosci.

If the filter *W*(*z*) has L-order transverse structure, therefore input signal *X*(*n*) of the filter *w*(*n*) can be described as

(4) $$\begin{array}{c} X\left(n\right)={\left[x\left(n\right),x\left(n-1\right),\ldots ,x\left(n-L+1\right)\right]}^{T}. \end{array}$$

The residual noise or error signal *e*(*n*) is given by

(5) $$\begin{array}{c} e\left(n\right)=d\left(n\right)-s\left(n\right)*\left[w{\left(n\right)}^{T}X\left(n\right)\right], \end{array}$$

where ^*∗*^ is the convolution sum.

Assuming that *M* is the length of the secondary path, then *E*[*e*^2^(*n*)] at the *n*th time is expressed by

(6) $$\begin{array}{c} E\left[e^{2}\left(n\right)\right]=E{\left[d\left(n\right)-\sum_{i=1}^{M-1}s_{i}\left(n\right)\sum_{j=1}^{N-1}w_{j}\left(n-i\right)\left(n-i-j\right)\right]}^{2}. \end{array}$$

We get the gradient of mean square error as follows:

(7) $$\begin{array}{c} \frac{\partial E\left[e^{2}\left(n\right)\right]}{\partial w\left(n\right)}=2e\left(n\right)\sum_{i=1}^{M-1}s_{i}\left(n\right)\frac{\partial x\left(n-i\right)}{\partial w\left(n\right)}, \end{array}$$

If the update step of weight coefficient is small enough, then

(8) $$\begin{array}{c} \frac{\partial J\left(n\right)}{\partial W\left(n\right)}=2e\left(n\right)x^{\prime }\left(n\right). \end{array}$$

The gradient descent algorithm of adaptive weighting coefficient is used in the ANC, so the weighting vector can be gained:

(9) $$\begin{array}{c} w\left(n+1\right)=w\left(n\right)+\mu e\left(n\right)X^{\prime }\left(n\right), \end{array}$$

where *μ* is the convergence factor. It affects convergence speed and stability in the FxLMS algorithm. To ensure stability, the convergence factor must be less than the maximum eigenvalue of the autocorrelation function.

The coefficient of the secondary path is determined according to the error signal during the convergence procedure. A trial-and-error process is used to make sure the factor emerges stable response, and it is slowly decreased until it emerges durable response.

Initially, ANC was used for a single channel, and later, it was extended to the multichannel. In comparison with single-channel noise suppression, the multichannel noise suppression has better performance to gain large quiet regions. Therefore, multichannel noise suppression based on the FxLMS algorithm is designed in this paper.

The article "Indoor Acoustic Signals Enhanced Algorithm and Visualization Analysis" was published in 2021. Journal: Comput Intell Neurosci.

In the FxLMS algorithm, the results of noise reduction under different parameters are obtained so as to further judge the best noise reduction performance. The antinoise signal is calculated as

(10) $$\begin{array}{c} G_{m}\left(k\right)=\sum_{j}Y_{m}^{\prime }\left(j\right)\varphi \left(k-j+1\right), \end{array}$$

where *Y*_*m*_′ is the control signal of the secondary path.

The signal received at the error microphone is

(11) $$\begin{array}{c} e_{m}\left(k\right)=d_{K}-G_{m}\left(k\right). \end{array}$$

The implementation of the ANC is defined as follows:

  Multichannel ANC includes one reference microphone, two control loudspeakers, and one error microphone
  Choose one acoustic sound position and three control positions

Figure 4 shows the error waveform in different received positions after and before ANC. At the same time, it shows the error waveform in different influence factors. The signal at the received position is consistent with the source signal at different positions. Meanwhile, variations of the signal at the received position are almost compatible with the source signal, except for some differences.

### 3.3. FCM Clustering Algorithm

FCM clustering is a flexible algorithm [35]. By calculating the membership matrix of the sample, the FCM clustering algorithm divides the objects into same-sized clusters with the greatest similarity and the different clusters with minor similarity. Although, in actual most cases, the dataset cannot be divided into distinctly separate clusters, assigning an object to a particular cluster can be rigid and can be error-prone. Therefore, it is better to use fuzzy c-means with natural, nonprobability characteristics in the FCM clustering algorithm.

Supposing the data are divided into *C* subsets, *C* centers of the subset are gained. Then, *u*_*ij*_ is the degree of membership that data *i* belongs to subset *j*. FCM clustering algorithm aims to find minimum value as following function [36, 37]:

(12) $$\begin{array}{c} J\left(U,c_{1},\ldots ,c_{C}\right)=\sum_{j=1}^{C}J_{j}=\sum_{j=1}^{C}\sum_{i=1}^{M}u_{ij}\left\|x_{i}-v_{j}^{2}\right\|, \end{array}$$

with the constraints:

(13) $$\begin{array}{c} \sum_{j=1}^{C}u_{ij}=1,\;\forall i;0\leq u_{ij}\leq 1,\forall j,\\ \sum_{i=1}^{M}u_{ij}>0,\;\forall i, \end{array}$$

where {*c*_1_,…, *c*_*C*_} is the set of clustering centers, ‖·‖ expresses the Euclidean distance, and *M* is the data length. Therefore, the equation can be solved by

(14) $$\begin{array}{c} u_{ij}=\frac{1}{\sum_{l=1}^{C}{\left(x_{i}-v_{j}/x_{i}-v_{l}\right)}^{\left(2/m-1\right)}},\;j=1,2,\ldots ,C;i=1,2,\ldots ,n,\\ v_{ij}=\frac{\sum_{i=1}^{M}u_{ij}^{m}x_{i}}{\sum_{i=l}^{n}u_{ij}^{m}},\;j=1,2,\ldots ,C, \end{array}$$

where *m* is the weighting exponent.

The article "Indoor Acoustic Signals Enhanced Algorithm and Visualization Analysis" was published in 2021. Journal: Comput Intell Neurosci.

## 4. Experimental Results

To validate the proposed method, we conducted an experiment to compare it with a baseline based on the LMS algorithm. Visualizations of sound field distributions are also presented to help to understand sound propagation. In addition, the FCM clustering algorithm is adopted to optimize the quiet points after indoor noise suppression.

### 4.1. Noise Inhibition

The two-way speaker noise control based on the FxLMS algorithm includes one noise source, one reference microphone, two antinoise loudspeakers, and one error microphone.

The ANC transfer function *P* (*z*) is

(15) $$\begin{array}{c} P\left(z\right)=0.01+0.25z^{-1}+0.5z^{-2}+z^{-3}+0.5z^{-4}+0.25z^{-5}+0.01z^{-6}. \end{array}$$

The secondary-path transfer function is defined as

(16) $$\begin{array}{c} S_{1}\left(z\right)=0.05-0.01z^{-1}+0.95z^{-2}+z^{-3}+0.9z^{-4},\\ S_{2}\left(z\right)=1+0.44z^{-1}-0.95z^{-2}+0.01z^{-3}+0.9z^{-4}. \end{array}$$

The 5 × 7 × 3 m^3^ room is the border of the indoor sound field. Its walls are not rigid in which absorption coefficient is 0.4. Figures 5(b)−5(c) show the noise inhibition results with LMS and FxLMS algorithms in the time domain, respectively. As we can see, both methods can reduce noise. In the beginning, the noise inhibition effect based on the FxLMS algorithm does not meet expectations. It is more significant with time increasing. The noise suppression based on the FxLMS algorithm is better than the system based on the LMS algorithm in the time domain.  Figure 5(d) shows the spectrum of original noise in the frequency domain.  Figure 5(e) describes the residual noise spectrum of the system based on the LMS algorithm.  Figure 5(f) describes the residual noise spectrum based on the FxLMS algorithm. The vertical axis denotes the noise amplitude after suppression in dB.  Figure 5 shows that the noise in the whole frequency band has been well suppressed. The system based on the FxLMS algorithm has a perfect suppression effect than based on the LMS algorithm.

Figure 6 depicts the experiment result of an 8 × 10 × 4 m^3^ medium-sized room, of which the impact factor *K* = 10 and the source position is [7.9, 9.9, 3.9]. The experiment result shows that the acoustic inhibition of the medium-sized room can reach 30 dB. Besides, the correlation between signal and interference is weak, and the reflection signal and refraction signal are not obvious for the large-sized room. The noise inhibition for the small-sized room is much more challenging, so the 5 × 7 × 3 m^3^ room is adopted in this paper.

### 4.2. Distribution of Sound Field

According to the sound field of the room, the acoustic vibration of each position at different times and spaces can be obtained. However, in the visualization stage, a large room will lead to difficulties for sound field simulation. Therefore, the room is divided into small units with 10 cm. Image sounds are used to simulate sound information at all the received positions.

The article "Indoor Acoustic Signals Enhanced Algorithm and Visualization Analysis" was published in 2021. Journal: Comput Intell Neurosci.

In the experiment, the positions of the noise source *r*_src_ and the reference microphone *r*_rmic_ are identical; both are [2.5 0.5 2] m. It is considered that the measuring height of the building is between 1.2 m and 1.5 m from the ground in the acoustic environment quality standard. Therefore 1.3 m is selected as the height in this paper, and the received position *r*_rmic_ is [2.5 5 1.3] m.

Considering the areas of human movement, we detect the areas between 1.0 m and 2.1 m in a vertical orientation. The amplitude ranges of [−0.001, 0.001] are defined as the quiet points. The acoustic distributions at times *t* = 0.03 s, 0.07 s, 0.4 s, and 0.6 s were examined to observe the sound propagation more intuitively.  Figure 7 shows the experiment results. Figures 7(b), 7(d), 7(f), and 7(h) show sound propagation at different times when the height *h* is 1.3 m.

Figure 7 depicts the direct sound signal that has not reached the received position at *t* = 0.03 s, which means there are many quiet regions in the room. At *t* = 0.07 s, the direct signal has nearly reached the received position. Some image signals have reached the received end at *t* = 0.4 *s* while the reverberation becomes more severe at *t* = 0.6 s.

### 4.3. Quiet Area Integration

The distribution density of quiet indoor points represents the comfort of certain areas in space. Because of the line of sight occlusion in three-dimensional space, it is difficult to distinguish the quiet local area with a concentration of points. The quiet local area can be represented intuitively through the quiet points' subdivision and the integration of the quiet areas.

After obtaining the quiet points, we adopt the Delaunay triangulation to subseparate the quiet points set. Firstly, it is integrated into two-dimensional space. During integration, specific spatial points can be integrated into the same point on the plane. As a result, not all the quiet points can be vertices of the Delaunay triangle.  Figure 8 shows the outcomes adopted by the Delaunay triangle and the quiet points at *t* = 0.03 s, 0.07 s, 0.4 s, and 0.6 s separately. It can be seen from the figures that there are a few quiet points in the space, but they still show a particular regional distribution. However, the quiet areas are larger than the others in Figure 8(a). Therefore, it would be convenient to integrate the quiet points set in the space directly. It is necessary to optimize the quiet point set to facilitate the description of the mute area.

The article "Indoor Acoustic Signals Enhanced Algorithm and Visualization Analysis" was published in 2021. Journal: Comput Intell Neurosci.

### 4.4. Optimization of the Quiet Areas

The quiet points obtained in the discrete acquisitions can either be distributed sparsely throughout the space or be grouped into distinct distribution groups. If we use the data to integrate the area directly, we can obtain nearly the whole area. However, as shown in Figure 8(g), there are only small quiet points. To tackle this issue, we use a FCM clustering algorithm to optimize all the quiet points before we integrate the Delaunay triangulation into the quiet area.

After the data are divided into *C* different subsets, the data are divided into different subsets to obtain an accurate quiet area. Quiet points are clustered with the FCM algorithm.

The quiet area in Figure 8 is not perfect when specific points are far away from the others. Furthermore, certain small areas contain many quiet points, whereas other regions have few quiet points. For this case, data with precise subcluster characteristics and continuity of volatility, the triangulation is obtained after separating the quiet points, and we segment the quiet points by the FCM clustering algorithm.

Figure 9 depicts the optimization results of the quiet area at different visual time points after the noise suppression through the combination of clustering algorithm and Delaunay triangulation. In Figure 9, the quiet area will be less as time increases, and it achieved good noise inhibition and has better than that without subset optimization.

## 5. Conclusions

In this paper, a multichannel ANC noise reduction method based on the FxLMS algorithm is realized in small-sized and medium-sized rooms. In addition, to illustrate and optimize the quiet areas in 3D indoor spaces, the combination of the FCM algorithm and Delaunay triangulation is also employed. The experimental results show that the proposed method of signal enhancement performs better than the system based on the LMS algorithm in noise inhibition. This is more conducive to examining the indoor effect and specific distribution of indoor noise reduction through visualization demonstration.

## Figures and Tables

**Figure 1:** The distribution of sound source and image source and received position in 3D space: (a) space structure of sound source point and received position and (b) the distribution of direct path and reflected path.

**Figure 2:** Impulse response on the different received positions *R*1, *R*2, *R*3: (a) *K* = 0, (b) *K* = 5, and (c) *K* = 15.

**Figure 3:** FxLMS algorithm block diagram.

The article "Indoor Acoustic Signals Enhanced Algorithm and Visualization Analysis" was published in 2021. Journal: Comput Intell Neurosci.

**Figure 4:** The noise reduction waveform of ANC at different received positions with *K* = 0, 5, and 15 in different rows, respectively. (a, d, g) The received position *R*1. (b, e, h) The received position *R*2. (c, f, i) The received position *R*3.

**Figure 5:** Acoustic inhibition comparison of the LMS and FxLMS algorithm. (a) Original noise in the time domain. (b) Residual noise in the time domain using the LMS algorithm. (c) Residual noise in the time domain using the FxLMS algorithm. (d) Original noise in the frequency domain. (e) Residual noise in the frequency domain using the LMS algorithm. (f) Residual noise in the frequency domain using the FxLMS algorithm.

**Figure 6:** Acoustic inhibition comparison based on FxLMS algorithm. (a) Original noise and residual noise in the time domain. (b) Original noise and residual noise in the frequency domain.

**Figure 7:** Indoor acoustic distributions in 3D space with different times: (a) *t* = 0.03 s, (c) *t* = 0.07 s, (e) *t* = 0.4 s, and (g) *t* = 0.6 s. Acoustic distributions at the height *h* = 1.3 m with different times of (b) 0.03 s, (d) 0.07 s, (f) 0.4 s, and (h) 0.6 s.

**Figure 8:** The distributions of quiet points at (a) *t* = 0.03 s, (c) *t* = 0.07 s, (e) *t* = 0.4 s, and (g) *t* = 0.6 s and their corresponding results after subseparation are shown in (b), (d), (f), and (h).

**Figure 9:** The quiet area distribution for the indoor environment after FCM algorithm with different times of (a) 0.03 s, (c) 0.07 s, (e) 0.4 s, and (g) 0.6 s at different rows, respectively, and their visualization results of using the FCM algorithm are shown in (b), (d), (f), and (h).

## Data Availability

The data that support the findings of this study are openly available and the details of source acoustic signal are provided in Section 3.1.
